# The Method of Pose Judgment of Potential Motion Damage in 3D Image Analysis

This article has been retracted.

**DOI:** 10.1155/2021/4743231

**Published:** 2021-11-29

**Authors:** Liping Gao

**Affiliations:** Sport College, Qujing Normal University, Qujing 655000, China

## Abstract

**Objective:**

This work aimed to study the posture judgment method of 3D image analysis of potential motion damage.

**Methods:**

The motion damage collection was implemented by the 3D image analysis method, and 3D image data were adopted to identify the motion damage data. Moreover, 3D image acquisition technology was adopted to analyze the model of potential motion damage and analyze the simulation judgment result of potential motion damage. Specifically, it included simulation parameters, motion damage posture collection effect, damage detection speed at the collection point, damage accuracy, and damage degree.

**Results:**

(1) The analysis of the damage monitoring speed at multiple collection points of the athletes in the sports environment confirmed that the range of changes in different time periods was different, and the changes showed a fast to slow to fast trend. (2) The 3D image analysis had high accuracy in analyzing the posture of potential motion damage, which rationalized the evolution of injuries. (3) The degree of motion damage under a 3D image changed from rising to gradual, which was in line with the theoretical results (all *p* < 0.05).

**Conclusion:**

3D image analysis can collect a high degree of small-sample-size data, then perform specific analysis, judgment, and summary, and finally, obtain objective and reasonable data. It greatly reduced the risk of potential motion damage for athletes and also improved the efficiency of injury recognition. Moreover, it reduced the chances of blind prevention and error prevention by athletes, thereby avoiding waste of resources. The simulation test confirmed the advantages of 3D image data collection in the sports environment, and it was solved that the current athletes cannot accurately and timely judge the potential motion damage. It also met the instability needs of the movement personnel of the acquisition system in the changing sports environment and provided a reliable guarantee for the safety and health of the sport personnel.

## 1. Introduction

Motion damage refers to the injury of the sports system that occurs during or during exercise. The human body's motion system includes bones, cartilage, joints, joint capsules, synovium, meniscus in joints, fish lips, and ligaments in joints. Any damage to these tissues, damage in activities, and sports are called motion damage [1]. At present, the overall condition of individuals in China is in a stage of continuous and rapid development. The health needs of society also put forward higher requirements for people's health. There are more and more potential injury problems caused by sports, and the judgment method has also received more attention [2].

Relevant researchers explored the correlation between psychological predictive factors such as the public fitness population's risk perception, risk taking, exercise ability judgment, motion damage experience, and motion damage from the perspective of sports psychology. Moreover, the predictive validity of these factors against motion damage in actual fitness exercises was measured, to provide a theoretical basis for further effective reduction and prevention of motion damage [3]. At present, research about potential motion damage is mainly posture research and to a certain extent, basic injury judgments in sports can be realized. In addition, most athletes can protect themselves and prevent themselves through injury prevention tutorials provided by coaches and other professionals [4]. However, since the current prevention tutorials for potential motion damage are not published, they are only provided for professional sports personnel, so comprehensive data information cannot be collected. Therefore, it is impossible to make accurate judgments, which hinders the preventive measures of potential injuries of athletes and also greatly wastes time and resources [5].

Modern motion damage is mostly chronic injuries with great hidden dangers. Two-dimensional image technology cannot accurately analyze and judge special parts. It is impossible to visually observe the evolution of the damage. It is also impossible to effectively distinguish the distribution of the internal medium space of the key parts during the movement, so that the final result does not have a large error in the actual damage part [6]. The 3D image can make up for the shortcomings of two-dimensional images. It can collect 3D images for potential damage caused by motion and then analyze and convert it into a motion model to facilitate the judgment of the result. The purpose of this research was exploring the 3D image analysis in pose judgment for potential motion damage. The report was as follows.

## 2. Motion Damage Collection Based on 3D Image Analysis

### 2.1. Motion Damage Collection with a 3D Image

The 3D image analysis method can distinguish three-dimensional moving images. Through the high-simulation of moving images, the noncommon extreme value of continuous images is discarded. The 3D image analysis introduced here recognizes and monitors continuous 3D images and realizes the simulation of continuous identification of 6 images at the same time. First, it is necessary to simulate and identify the structure of the movement. Then, specific motion set parameters and two-dimensional motion images are adopted to analyze the 3D image features. It is assumed that the component matrix after the known multidimensional motion characteristics has passed the damage identification as follows:

(1) $$\begin{array}{c} Z=\left\{u_{1},\ldots ,u_{n}\right\}. \end{array}$$

The damage process determined by a 3D image is as follows:

(2) $$\begin{array}{c} Z_{i}=\left\{\begin{array}{c} u_{1}{\;}_{i}\\ r_{i}\\ \ldots \\ u_{ni}\\ r_{ni} \end{array}\right\}. \end{array}$$

In equation (2), *Z*_*i*_ represents the feature point of the *i*-th injury after motion damage and *n* represents the *n*-th frames of each moving image.

The motion damage posture acquisition method based on 3D image analysis uses equation (3) to mark the constructed 3D injury image for point damage. After the matrix of the motion structure is replaced, the transformed high-order matrix is obtained, as shown in equation (4).

(3) $$\begin{array}{c} Z_{i}=\left\{\begin{array}{c} u_{1i}r_{1i}s_{1i}\\ \ldots \\ u_{ni}r_{ni}s_{ni} \end{array}\right\}. \end{array}$$

(4) $$\begin{array}{c} Q_{i}=\left\{\begin{array}{c} u_{1i}\\ r_{1i}\\ \ldots \\ u_{ni}\\ r_{ni} \end{array}\right\}. \end{array}$$

In the function, the difference between *Z*_*i*_ and *Q*_*i*_ can be expressed as the *WT*_*4*_ incidence matrix, and two matrices were adopted for fusion conversion.

(5) $$\begin{array}{c} {\text{WT}}_{4}=Z_{i}-Q_{i}=\left[\text{quater}\left(n\right)\right]\left[\text{quater}\left(n\right)*Z_{i}+Q_{i}\right]-Z_{i}. \end{array}$$

The final result can help realize the recognition of multi-image motion damage.

### 2.2. Posture Acquisition for Motion Damage

To utilize 3D image data to identify the injury data of the athlete, it is necessary to mark and confirm the injury part through the 3D image. However, the introduction of the abovementioned 3D image analysis method is still unable to judge in the completed collection of damage data. Assuming that the damage data of the 3D sports damage image is *A (m, n)* and the damage posture is represented by *p* *+* *l*, the damage matrix formula *S* is as follows:

(6) $$\begin{array}{c} S_{pl}=\sum_{m}\sum_{n}\left(m-\bar{m}\right)\left(n-\bar{n}\right)\left(mn\right). \end{array}$$

Since the shooting angles of the obtained 3D motion images are different, the clarity of the image needs to be processed. To avoid image interference and data shock, the posture of the data must be transformed. The formula of *E*_*pl*_ is as follows:

(7) $$\begin{array}{c} E_{\text{pl}}=\text{spl}\left(s_{p}^{2}-s_{l}^{2}\right)-s\left(s_{l}^{p}s_{p}-s_{l}^{p}s_{l}\right). \end{array}$$

Through the 3D damage matrix and the change of the damage image display, the specific data of the athlete's injury *s*_*p*_^2^ is obtained, and *s*_*l*_^2^*y* is the related parameter of the injury, which can realize the data positioning of the posture.

The abovementioned damage data can be restricted in the motion structure matrix and can be extracted by calculating the variance. If the variance is less than the hypothetical value in the theory, it can be replaced with a theoretical value for extraction. The realization process of the motion damage posture acquisition method based on 3D image analysis designed in this research is shown in Figure 1.

## 3. Potential Motion Damage Posture Judgment Simulation Based on 3D Image Analysis

### 3.1. Analysis of 3D Image Acquisition Technology

With the development of science and technology, computer technology and computer graphics have been rapidly developed, and the application range of 3D image display technology has become more and more extensive. Due to various uncertain factors from the outside world, the human organs are destroyed anatomically or functionally, causing varying degrees of local or systemic damage. The collection of 3D images can facilitate the judgment of damage during exercise, and the accuracy of image collection directly affects the correctness of damage judgment. 3D image acquisition is the adoption of a computer to develop the presented graphics and model library into a graphics standard that can be shared and then take it as the acquisition standard. This technology is different from hardware and window systems, which can work independently in a network environment. Then, it is presented as standard graphics in high-end applications such as professional graphics processing and scientific computing.

### 3.2. Establishment of a Model of Potential Motion Damage

Due to the relatively stricter life rules of athletes, they are also restricted to a certain extent. In addition, the physical load of athletes with lower physical fitness is too large, and they are prone to disorder of movement rhythm, which can eventually cause the body to be often in a state of fatigue. As a result, the accuracy of the movement and the reduction of athletic ability appear, and even alertness and concentration are reduced. The model of motion damage is shown in Figure 2.

When the athlete is doing strong exercise, the metabolism of the individual is strong, and the lactic acid also accumulates in a large amount. The elasticity of muscles and ligaments, the coordination of antagonistic muscle groups, and the flexibility of joints are all weakened to varying degrees, which easily lead to serious motion damage during sports. Therefore, it is particularly important to take preventive measures for sports personnel, so as to judge potential injuries according to the sports personnel's own conditions.

## 4. Simulation Analysis of the Posture of Potential Motion Damage

The 3D image acquisition method under the motion state was simulated into the system for judging potential motion damage. A certain athlete was taken as a test case to construct his sports environment, and 3D image acquisition parameters were set, respectively. The posture judgment of potential motion damage based on 3D image analysis was simulated, and the parameters of the simulation were set as shown in Table 1. The effects of motion damage posture acquisition, the speed of injury detection at the acquisition point, the accuracy of injury, and the degree of injury were analyzed, respectively.

### 4.1. Simulation Parameter Value Setting

#### 4.1.1. Analysis of Sampling Points

*(1) Motion Damage Posture Collection Effect (Take a Specific Sport as an Example)*.  Figure 3 showed that the long-term maintenance of a specific posture during exercise would cause permanent damage to a certain part of the body.

*(2) Analysis of the Damage Detection Speed of the Collection Point*. The damage monitoring speed at multiple collection points of athletes in the sports environment was analyzed as shown in Figure 4, it was found that there are differences in the range of changes in different time periods, and the changes showed a fast to slow to fast trend, with a considerable difference (*p* < 0.05).

*(3) Damage Accuracy Analysis of the Collection Point*. The results showed that the 3D image analysis of potential motion damage poses was more accurate as shown in Figure 5, which rationalized the evolution of the injury, and the difference was statistically considerable (*p* < 0.05).

*(4) Analysis of the Damage Degree of the Collection Point*. The results showed that the degree of motion damage under a 3D image changed from rising to gradual as shown in Figure 6, which was consistent with common sense, and the difference was statistically substantial (*p* < 0.05).

## 5. Conclusions

Based on 3D image analysis, the simulation of the posture judgment of potential motion damage showed the motion damage data more comprehensively. Compared with the shortcomings of traditional motion damage judgment, it can increase the inertia of the movement of the vulnerable parts of the injury, making the entire judgment process of injury more realistic [7]. The results revealed that the analysis of the damage monitoring speed of the athletes in the sports environment at multiple collection points confirmed that the range of change in different time periods was different, and the change showed a fast to slow to fast trend. Moreover, the accuracy of the posture of potential motion damage analyzed by a 3D image was high, which rationalized the evolution of injuries. In addition, the degree of motion damage under a 3D image had changed from rising to smooth, which was consistent with common sense. These results all reflected the accuracy of a 3D image in judging potential motion damage, which were consistent with the results of most researchers.

For traditional analysis, the collection of damage data is difficult, resulting in incomplete data services, and it is limited to the prevention of damage under the knowledge of professionals. The research of a 3D image can collect a high degree of small-sample-size data [8]. Then, specific analysis, judgment, and summary were made, and finally, objective and reasonable data were acquired. It greatly reduced the risk of potential motion damage for athletes and improved the efficiency of injury recognition. Furthermore, it reduced the chance of blind prevention and error prevention by athletes, thereby avoiding waste of resources [9].

The simulation test used in this research was one of the important processes of the 3D image analysis of the judgment method of potential motion damage. The simulation test confirmed the advantages of 3D image data collection in the sports environment and solved the problem of inaccurate and timely judgment in the existing potential motion damage of sports personnel [10]. It also met the instability needs of the movement personnel of the acquisition system in the changing sports environment and provided a reliable guarantee for the safety and health of the movement personnel.

The shortcoming of this research is that it does not show the research process of a 3D image in detail, so further research and investigation are needed, so as to get practical and reliable research data results.

## Figures and Tables

**Figure 1:** A method for acquiring motion damage posture based on 3D image analysis.

**Figure 2:** Schematic diagram of the athlete's potential injury model.

**Figure 3:** The effect of motion damage posture acquisition.

**Figure 4:** Damage detection speed at the collection point.

**Figure 5:** Damage judgment accuracy of the collection point.

**Figure 6:** Damage degree of the collection point.

**Table 1:** Simulation parameter value setting.

Parameter	Set value
Degree of damage during sport	Below grade 4 damage
Relative muscle exercise	45% or more
Simulation image floating value	(−13, 55)
Exercise interval	15s
Number of simulations	800
Simulation duration	20 min

## Data Availability

The data used to support the findings of this study are available from the corresponding author upon request.
